# Microcytic and Malarial Anaemia Prevalence in Urban Children ≤15 Years in the Mount Cameroon Area: A Cross-Sectional Study on Risk Factors

**DOI:** 10.1155/2021/5712309

**Published:** 2021-04-08

**Authors:** Sharon Odmia Sama, Seraphine Njuontsop Chiamo, Germain Sotoing Taiwe, Gwendolyne Elobe Njume, Irene Ule Ngole Sumbele

**Affiliations:** ^1^Department of Zoology and Animal Physiology, University of Buea, Buea, Cameroon; ^2^Department of Microbiology and Immunology, Cornell College of Veterinary Medicine, Ithaca, NY, USA

## Abstract

**Background:**

Anaemia, a common nutritional deficiency, is a public health problem in the Mount Cameroon area. This study determined the prevalence and possible risk factors of microcytic and malarial anaemia in children less than ≤15 years residing in the Buea and Limbe municipalities in the Mount Cameroon area.

**Methods:**

A total of 566 children were clinically examined in a cross-sectional study from December 2018 to August 2019 for anaemia and malaria parasites. Blood samples collected were used in evaluating full blood count with the aid of an automated haemoanalyser, and malaria parasite was confirmed by microscopy. Anaemia was defined based on WHO standards while microcytic anaemia and malarial anaemia were defined as microcytosis + anaemia and malaria + anaemia, respectively. Factors that showed significance in the bivariate analysis were entered into a multinomial logistic regression to determine risk factors for microcytic and malarial anaemia.

**Results:**

The overall prevalence for anaemia, microcytosis, microcytic anaemia, and malarial anaemia was, respectively, 68.7%, 48.9%, 36.9%, and 19.6% with microcytic anaemia representing 53.7% of all anaemic cases. Risk factors for microcytic anaemia included child age of 1–5 years (*P*=0.007), forest ethnicity (*P*=0.019), parents being farmers (*P*=0.038) or jobless (*P*=0.009), and having moderate malaria parasitaemia (*P*=0.048) while those for malarial anaemia were child age of 6–10 years (*P*=0.008), parents' age of 26–35 years (*P*=0.049), parents being jobless (*P*=0.023), and consuming plantains 3-4 times (*P*=0.024) a week.

**Conclusion:**

Microcytic anaemia is getting to be a severe public health concern while malarial anaemia is a mild public health issue in children residing in urban areas of Mount Cameroon. Parents' occupation was directly linked to all anaemia forms; hence, any intervention to curb anaemia should consider aspects that will raise the socioeconomic status of the population.

## 1. Introduction

Anaemia is still a public health problem in developing countries [1] across all age groups [2]. It is a condition where blood haemoglobin concentration is lower than the normal for a person's age, gender, and environment [3, 4]. Notably pregnant women, and children because of rapid development and impact on cognitive development, are most at risk of anaemia. The adverse health consequences and impact are felt at both the individual and societal levels [5–8]. Globally, anaemia prevalence stands at around 2 billion with over 800 million anaemic children and women; Africa and Asia bear the brunt with an estimated 85% prevalence [5]. In Cameroon, as in the Mount Cameroon area, anaemia is still a severe public health problem. Most recent estimates from the World Bank show a prevalence of 62.5% in children under five and 49.3% in pregnant women [9].

Anaemia is not a standalone condition but results from lack of one or more micronutrients, infections such as malaria and hookworm, congenital haemolytic diseases, poor maternal health, socioeconomic status, and even demographic factors [10–12]. Malaria is often associated with anaemia and is a major contributor to the occurrence and severity of anaemia in malaria endemic zones. Its route of action is seen in the destruction of both parasitized and nonparasitized red cells [13]. The parasites feed on host haemoglobin, and to stop them from acquiring host iron, the recycling of iron by reticuloendothelial (RE) macrophages is impeded [14, 15]. This leads to lack of iron in the cell that may ultimately lead to iron deficiency (ID) and consequently microcytic red cells and anaemia.

Microcytic anaemia which is characterised by smaller than normal circulating red blood cell for age [16] is a common type of anaemia. While iron deficiency is the main cause of microcytic anaemia, thalassaemia trait (which is a defect in haemoglobin synthesis), chronic inflammation (resulting from lack of iron), and other haemoglobinopathies (such as sideroblastic anaemia) are implicated [17]. Microcytic anaemia often goes undetected except incidentally encountered when full blood count is run for other reasons [18], hence, the need for regular monitoring of its occurrence. Another anaemia type of common occurrence is iron deficiency anaemia (IDA) which results from depleted iron stores due to poor absorption or poor or reduced iron intake and poor erythropoiesis [19]. However, a person can be functionally iron deficient without out-rightly manifesting anaemia as often seen in mild to severe anaemia. Nonetheless, as IDA worsens, the red cells of its victims are exposed to oxidation and reduced antioxidant defence [20].

While several studies in the Mount Cameroon area have determined the occurrence of anaemia in conjunction with malaria and other infections in various setting, the type of anaemia which is invaluable in making informed decision when planning control measures has been infrequently examined. Therefore, the objective of this study was to determine the prevalence and identify factors associated with microcytic and malarial anaemia in children ≤15 years living in urban areas of Buea and Limbe in the Mount Cameroon area.

## 2. Methods

### 2.1. Study Sites and Participants

The study was conducted in the Buea and Limbe I and III municipalities, both located in the Mount Cameroon area of Fako Division. Buea is situated and characterised as described by previous studies [21]. It is divided into 7 health areas, namely, Bokwango, Bova, Buea Road, Buea Town, Molyko, Muea, and Tole. Limbe has been described by previous studies [22]. In terms of health areas, the Limbe Health District is subdivided further into 8 health areas, namely, Batoke, Bimbia, Bojongo, Bota, Mabeta, Moliwe, Limbe Regional Hospital, and Sanje. These 8 health areas fall under 3 councils: Limbe I (Poh), Limbe II, and Limbe III councils. Malaria parasite transmission in Cameroon is very heterogenous varying with altitude and climate [23]. In the Mount Cameroon area, transmission is holoendemic and perennial with lower altitudes having the highest transmission rates [24]. Entomological inoculation rates (EIR) reported in the area before vector control measures were implemented ranged from 149.0 to 287.0 infectious bites per person per year (ib/p/y) in coastal towns like Limbe, Tiko, and Idenau [25]. This rate witnessed a drop to 0.7–1.4 ib/p/m [26] after the use of long-lasting insecticide-treated bed nets (LLINs) was implemented.

The study population included children 1–15 years living in the study area whose parents or caregivers gave consent to their participation in the study. Those with known HIV status, with active haemorrhage, who had blood transfusion or were operated upon two months prior to the study, and who are or had been on antimalarials two weeks prior to the study were excluded.

### 2.2. Study Design, Sampling Technique, and Unit

This cross-sectional study was carried out from December 2018 to August 2019. Following administrative and ethical clearances, participants were enrolled into the study at their various communities and at presentation to the hospital following education. Informed consent/assent forms were given to parents/caregivers explaining the purpose, benefits, and risks of the study. Structured questionnaires to obtain information on sociodemographic data, type of accommodation, clinical history, and dietary habits were administered, and clinical evaluation and blood samples were collected thereafter for malaria parasite determination and full blood count (FBC) analyses.

A convenient multistage sampling method was employed in the study. Firstly, for representativeness of each health district, a health area was randomly selected from each of the 3 council areas that make up the Limbe Health District and 2 were selected from the 4 distinct urban settings recognised in the Buea Health District. This was followed by a random selection of representative health facilities and neighbourhoods in the selected health areas. Following education by the community relay agents, potential participants in the selected communities were invited to a specified data collection hall in the neighbourhood on programmed dates coordinated by the neighbourhood head. Concurrently, at presentation to the outpatient department of both Buea Regional and Bota District Hospitals, participants were enrolled prospectively as they fulfilled the inclusion criteria for the study. The sample size for the study was determined using the formula *n* *=* *z*^2^*pq*/*d*^2^ [27], where *n* was the required sample size; *z* was 1.96, the standard deviation for a 95% confidence interval (CI); *P* value was 62% which was the anaemia prevalence in the region [21]; *q* was (1 − *p*); and *d* was the acceptable error margin set at 0.05. The optimum sample size for both health districts was 362. To allow for data loss due to incomplete data entry, the sample size was increased by 10% to 400 requiring an average of 200 samples per health district.

### 2.3. Data Collection

Each child was examined clinically by a trained physician. With the assistance of an interviewer, the parent/caregiver was given a self-administered structured questionnaire to fill, and this included information on sociodemography, clinical symptoms, type of habitation, and dietary habits. Axillary temperature was measured using a clinical thermometer, and fever was defined as temperature ≥37.5°C. Symptoms such as cough, headache, diarrhoea, and body weakness/pain were recorded. Weight and height were measured using a Terraillon weighing scale and a measuring tape to the nearest 0.1 kg and 1 cm, respectively. Parents of children who could not walk were requested to climb on the balance with the child and then without the child; the difference between both weights was recorded as the child's weight. The recumbent length was measured for children who could not walk. Height-for-age (HA), weight-for-age (WA), and weight-for-height (WH) z-scores were computed based on WHO growth curves [28] using WHO Anthro and AnthroPlus packages [29]. Stunting, underweight, and wasting were, respectively, defined as HA, WA, and WH *z*-scores of <−2. Malnutrition was defined as any *z*-score <−2 [16]. Dietary assessment was done by a recall by parents on how often in a week they consumed the following foods: fruits, vegetables, meat, fish, and plantains. This was scored as (1) 1-2 times, (2) 3-4 times, and (3) >4 times a week.

### 2.4. Laboratory Methods

Approximately 4 mL of venous blood was collected using sterile techniques into EDTA and dry tubes. Labelled blood samples were transported on ice to the Malaria Research Laboratory of the University of Buea for further analysis. Thin and thick blood films were prepared immediately after dispensing blood into EDTA tubes. Thin films were fixed with absolute methanol and together with the thick films stained for 15 minutes with 10% Giemsa stain and then examined for the detection and identification of the malaria parasite following standard procedures [30]. Slides were considered positive when asexual/gametocyte forms were observed, and parasitaemia was calculated per 200 white cells multiplied by patient's white blood cell (WBC) counts and stretched to 500 leukocytes if gametocytes were seen [30]. Parasite burden was classified per microliter (*μ*L) of blood as low (<1000 parasites), moderate (1000–4999 parasites), high (5000–99,999 parasites), and hyper (≥100,000 parasites) [31].

Blood in the dry tube was centrifuged at 3000 rpm for 5 minutes, and the aliquots were stored at −20°C until use. C-reactive protein (CRP) concentration was determined using the Thermo Fisher ELISA machine as per the manufacturer's instructions. Inflammation was confirmed when acute phase protein (APP) CRP was >5 mg/L [20]. A complete blood count was run using the Nihon Kohden Celltac *α* haemoanalyser according to manufacturer's instructions to obtain values for WBC, red blood cell (RBC) and platelet (Plt) counts, haemoglobin (Hb), haematocrit (Hct), mean cell volume (MCV), mean cell haemoglobin (MCH), mean cell haemoglobin concentration (MCHC), red cell distribution width coefficient of variation (RDW-CV), red cell distribution width standard deviation (RDW-SD), mean platelet volume (MPV), and platelet distribution width (PDW). Anaemia was classified based on WHO age-based classification [32] as Hb < 11.0 g/L for children 1–5 years, Hb < 11.5 g/dL for children 6–11 years, and Hb < 12.0 g/dL for children 12–15 years old. Severe anaemia was defined as Hb < 7.0 g/dL for all children. Moderate anaemia was defined as Hb: 7.0–9.9 g/dL for 1–5 years and Hb: 7.0–10.9 g/dL for children 6–15 years, and mild anaemia was defined as Hb: 10.0–10.9 g/dL for children 1–5 years, Hb: 11.0–11.4 g/dL for children 6–11 years, and Hb: 11.0–11.9 g/dL for children 12–15 years. Malaria anaemia (MA) was defined as anaemia + positive blood smear for malaria parasite while nonmalarial anaemia (NMA) was defined as anaemia with negative blood smear for malaria parasites. Microcytosis was defined as MCV <67 fL for children less than 2 years and MCV <73 fL for children 2 to 15 years, and microcytic anaemia was defined as Hb < 11.0 g/dL + MCV< 67 fL and Hb < 11.0 g/dL + MCV <73 fL, respectively [16].

### 2.5. Data Analysis

Data was keyed into Microsoft Excel 2010 and exported into IBM-Statistical Package for Social Sciences (SPSS) version 20 (SPSS, Inc., Chicago, IL, USA). Continuous variables were summarized as means and standard deviations while categorical variables were reported as percentages and frequencies. Proportion difference was evaluated using Pearson's Chi square test (*χ*^2^), Pearson's ranked correlation (*r*) for haematological bivariate association, and analysis of variance (ANOVA) to compare group means. Parasite density was log-transformed before analysis. Factors with a *P* value <0.2 in the bivariate analysis were entered into a multinomial logistic regression to determine risk factors for microcytic and malarial anaemia. Odd ratios (OR) and 95% confidence intervals (CIs) were computed, and *P* < 0.05 value was suggestive of statistical significance.

### 2.6. Ethical Consideration

Ethical clearance was obtained from the Institutional Review Board hosted by the Faculty of Health Sciences, University of Buea (2018/811–05/UB/SG/IRB/FHS), following an administrative approval from the Regional Delegation of Public Health (R11/MINSANTE/SWR/RDPH/PS/430/940). Authorisations from community heads were also obtained. Only children whose parents consented to their participation in the study and who responded to the questionnaires were enrolled after the purpose, risks, and benefits were clearly explained to them. It was stressed that the study was completely voluntary and that a parent had every right to stop/withdraw their child from the study. Even after the parent's consent to participate in the study, any child who was too scared of a needle was not forced to continue. Data was treated with utmost confidentiality by assigning codes to the patients' samples.

## 3. Results

### 3.1. Baseline Characteristics of Study Participants

A total of 614 participants were approached to participate in the study, and 589 of them were enrolled. After data curation, 566 participants were retained of which 47.2% were males and 52.8% were females, living in low (61.5%) and highland (38.5%) areas. The mean (SD) age was 6.4 (4.5) years of whom 51.4% were ≤5 years. As shown in Table 1, most of the participants were enrolled at presentation to hospital (63.3%), had household head between 35 and 50 years old (44.2%), and had secondary level of education (40.6%). Overall, anaemia, malaria, microcytosis, inflammation, fever, and malnutrition prevalence in the study population were, respectively, 62.4%, 27.7%, 48.9%, 58.4%, 27.7%, and 15.2%.

### 3.2. Malaria Parasite, Nutritional Status, and Dietary Habits

Significantly higher prevalence of malaria parasite was observed in children aged 6–10 years (35.5%, *P*=0.003), those from low altitude (32.8%, *P*=0.001), and those who presented themselves at the hospital (33.5%, *P* < 0.001) when compared with their respective contemporaries. The prevalence of malaria parasite and malnutrition was comparable with sex (*P*=0.715 and *P*=0.421, respectively). However, significantly higher occurrence of malnutrition was observed in children aged 1–5 years (21.0%; *P* < 0.001), those living at low altitude (18.1%; *P*=0.015), those whose parents were fishermen (23.3%, *P*=0.025), and those of other ethnicity (26.5%; *P*=0.029) as shown in Table 2.

On dietary habits, more children ≤5 years reported not washing hands before meals (19.9%) and consuming fewer plantain meals a week than their older peers. This difference was statistically significant (*P*=0.001 and *P*=0.038, respectively). The weekly plantain consumption was significantly linked to parents' education level (*P*=0.049) with more children whose parents had no formal education consuming plantain ≥3 times weekly (55.8%) when compared with their counterparts as shown in Figure 1.

### 3.3. Anaemia, Microcytic Anaemia, and Malarial Anaemia Prevalence

Overall, the prevalence of anaemia (68.7%) was highest in children living in low altitude (77.3%), examined in the community (81.2%), and living in homes with 6–10 occupants (71.4%) and whose parents were 25–35 years old (80.2%), had no formal education (75.8%), or were fishermen (86.4%) as well as those of forest ethnicity (100.0%) when compared with their compeers. The differences were statistically significant. In relation to clinical factors, the only significantly higher prevalence of anaemia (*P*=0.011) was observed in those with inflammation (79.1%) as shown in Table 3.

The prevalence of microcytic anaemia was 36.9% accounting for 53.7% of all the anaemic cases. Significantly, it was highest in children ≤5 years old (43.3%), those living in low altitude (49.1%), those examined within the community (42.8%), those whose parents were 26–35 years old (39.7%) and were fishermen (56.3%), those of forest ethnicity (60.0%), those malaria parasite positive (49.7%), and those who had moderate parasitaemia (62.8%) when compared with their respective contemporaries. While malarial anaemia occurred in 19.6% of the study population, children aged 6–10 years (24.1%), those living at low altitude (23.9%), those whose parents were 26–35 years old (21.6%), and those who were feverish (28.7%) and were malaria parasite positive (68.8%) had significantly higher prevalence than their respective peers (Table 3).

### 3.4. Effect of Nutritional Status and Dietary Habits on the Different Types of Anaemia

The prevalence of anaemia was significantly higher (*P*=0.010, *P*=0.047, and *P*=0.009) in children who were stunted (83.1%), were underweight (89.5%), and consumed plantains 3-4 times a week (85.3%), respectively, when compared with their equivalents. On the other hand, microcytic anaemia prevalence was significantly higher (*P*=0.048) in normal (43.7%) than wasted children, while only those who consumed plantains 3-4 times a week had a significantly higher (*P*=0.025) prevalence of malarial anaemia (20.6%) as shown in Table 4.

### 3.5. Risk Factors for Anaemia, Microcytic Anaemia, and Malarial Anaemia

As revealed in Table 5, the logistic regression analysis with anaemia as dependent variable showed that children living in lowland (*P*=0.017), those whose parents were farmers, worked privately, or were fishermen (*P*=0.042;*P*=0.013;*P* < 0.001, respectively ), and those who consumed meat 3-4 times weekly (*P*=0.026) and plantains (*P*=0.034) were significantly at risk of developing anaemia. They were, respectively, 4, 2.2, 2.7, 5.5, 2.5 and 2.5 times more likely to be anaemic than their counterparts. Significantly, children aged 1–5 years (*P*=0.007), those of forest ethnicity (*P*=0.007), those whose parents are farmers (*P*=0.038) or jobless (*P*=0.009), and those who had moderate parasitaemia (*P*=0.048) were 2.4, 15.7, 2.5, 3.4, and 2.6 times, respectively, more likely to have microcytic anaemia. With respect to malarial anaemia, the identified risk factors were the child's age (*P*=0.008), parent's age (*P*=0.049) and occupation (*P*=0.023), and child's weekly consumption of plantain (*P*=0.024). Children aged 6–10 years, whose parents were 26–35 years old or jobless, and who consumed plantains 3-4 times a week were 3.3, 2.6, 3.8, and 2.9 times, respectively, more likely to have malarial anaemia than their counterparts.

## 4. Discussion

This study investigates the prevalence and risk factors for microcytic and malarial anaemia in children 1–15 years in urban settings of the Mount Cameroon area. The overall malaria prevalence of 27.7% is like that reported by Teh et al. [33] with the highest burden (35.5%) observed in children in the 6–10 years age group and those living in low altitude. The shift in malaria burden from the under-fives to the 6–10 years observed in this study may be due to effective bed net use in the former corroborating findings elsewhere [34].

More than half of the study participants reported washing hands before meal and consuming plantains more than twice weekly. Hand washing increased with age because younger children must be reminded frequently to wash their hands but will form the habit as they grow older. This finding is corroborated by studies elsewhere [35]. In addition, findings from the study revealed that plantain consumption increased with child's age but decreased with parent's level of education. Younger children may prefer the ripe version of the plantain or paste, which is easier for them to chew/swallow but contains more carbohydrates, to the harder unripe plantain [36] consumed easily by older children which has more of iron and vitamin C. On the other hand, increase in the level of schooling increases knowledge on better feeding practices and dietary diversity [37, 38]; also income may account for the decrease in plantain consumption with rise in level of education as participants can probably afford to replace plantains with other iron-rich foods. That notwithstanding, unripe plantains are rich in iron and vitamin C which are two micronutrients that optimize absorption and can aid in avoiding the occurrence of anaemia [39].

The overall anaemia prevalence of 68.7% reveals that anaemia is a serious public health problem in children in this region as elsewhere in the country. This is higher than both the national anaemia prevalence of 60% [9] and that observed by Teh et al. [34] in the same area but lower than the 77.2% reported in Tanzania [111]. The higher prevalence of anaemia among the 6–10 years old compared with their counterparts is not a surprise as a similar higher prevalence of malaria was observed in the same group. Malaria parasite infection has been reported severally as a risk factor of anaemia [21, 22, 34]. In addition, observations from studies in the Mount Cameroon area have revealed that the burden of malaria has shifted from the ≤5 years old to older age groups due to the increased preventive measures in the former group [34, 40, 41]. This age-related change in burden of malaria may have led to the shift in anaemia prevalence from the under-fives to older groups.

That anaemia was more prevalent at lower (Limbe municipality) than higher altitude (Buea municipality) in this study shows the association between malaria, anaemia, and altitude which had long been established in previous studies [11, 33, 42]. Children living at lower altitude were 4 times at odds of being anaemic. Higher temperatures at low altitudes favour breeding of the malaria vector and transmission of malaria parasites [43–45] which in turn leads to increased anaemia prevalence as malaria has been shown to be among the major contributors to the occurrence of anaemia in this setting [34].

Contrary to findings by Sakwe et al. [45] who reported lower anaemia prevalence in a community-based study than in sick children seeking treatment in the hospital, our findings revealed that anaemia was more present in children within the community than at presentation to hospital. This may be due in part to the occurrence of submicroscopic *Plasmodium* infection that was not determined and the prevalence of malaria parasite observed in these apparently healthy children in the community. It is established that malaria causes haemolysis of both parasitized and healthy red cells leading to anaemia [13]. Also, in malaria parasite intense transmission regions, apparently healthy children may have subclinical infection even in the absence of overt disease. Effect of these subclinical infections are usually determined by measuring the concentration of acute phase proteins such as CRP involved in the inflammatory response. Inflammation being primarily protective [46] also causes the retention of iron by the reticuloendothelial macrophages leading to lower iron concentration in circulation and thus anaemia [47].

Parents' age, education level, occupation, and ethnicity as well as family size are sociodemographic factors that are intrinsically linked and significantly associated with childhood anaemia as reported in previous studies [38, 48, 49]. Parents who were ≤35 years old and those with no formal education had more anaemic children than the other parents. Being ≤25 years old may suggest that as first-time parents they are less prepared for parenthood and meeting the nutritional needs of the child. This may also be compounded by lack of knowledge on childcare and anaemia [50, 51]. Also, because a parent has little or no formal education, their chances of getting skilled jobs are also very reduced, leading to low wages and limited access to healthy food sources [52]. The odds of having anaemia was lesser in children in homes with >10 occupants. Contrary to studies where people living in or in proximity to forested areas have normal haemoglobin levels [53], findings from this study reveal that children with forest origin had the highest prevalence of anaemia. It may be that being away from their area of origin keeps them away from wild game and diverse forest foods which have been shown to improve iron intake and limit anaemia [54, 55].

Although not significant, observations from this study reveal that children who were feverish, were malaria parasite positive, and had moderate parasitaemia were more anaemic than their respective counterparts supporting findings from elsewhere [30, 56]. Fever is known as a characteristic symptom of malaria even though nonspecific where other infections are possible [57]. The fever may have been caused by immune responses to malaria or some other underlying disease.

Malnutrition affects all strata of the society but mostly children are more vulnerable because of high nutritional demands required for proper growth [58]. Anaemia was more common in malnourished children and was significantly higher in stunted (83.1%) and underweight (89.5%) children than their counterparts. This finding is in line with studies carried out in Bangladesh by Rahman et al. [59]. However, nutritional deficiencies may not always be directly linked to anaemia but could be the cause that weakens the general health of the children exposing them to other anaemia-causing diseases. This is supported by Khanam et al. [60].

Regarding microcytosis and microcytic anaemia, an overall 48.9% of the study population had microcytosis while microcytic anaemia prevalence was 36.7%. This proportion ranks it as a moderate public health concern according to WHO classification on anaemia burden [32]. This proportion of 36.7% is comparable to that observed in Tanzania [11] but lower than the 49.0% observed by Mah et al. [40] in children seeking treatment in the Yaounde Gynaeco-Obstetric and Paedriatric Hospital. Microcytosis is defined as a lower than normal MCV for age. It is indicative of iron deficiency, and iron deficiency is said to be responsible for half of all anaemia cases [61]. However, since we did not measure ferritin levels and other markers for iron status, we may have underestimated the true depiction of iron deficiency in the population.

Males had higher microcytic anaemia prevalence (70%) than females although this observation may not be a surprise since the males equally had higher prevalence of malaria and anaemia than females. Age-wise, we would have expected children 6–10 years old to have the highest prevalence of microcytic anaemia as with both malaria and anaemia but that was not the case. Instead, the ≤5 years old had significantly higher prevalence of microcytic anaemia than their counterparts. Microcytosis and anaemia each have varied aetiologies, the result of which in combination may lead to microcytic anaemia. The observed microcytic anaemia in this case may have been due to anaemia resulting from nutritional deficiency and not malaria, as children in this age have high iron needs for growth. Furthermore, microcytosis may have been due to the body's protective mechanism to wade off infection with malaria parasite [62], or resulting from some other anaemia-causing factor such as the thalassaemia trait, a common haemoglobinopathy in malaria endemic African populations. It may also result from bacterial, viral, or helminth infections which were not evaluated, as it was out of the scope of this investigation and thus a probable limitation of the study.

A significant association between occupation, ethnicity, and microcytic anaemia is like that observed with anaemia. Parents who were jobless, fishermen, and farmers had children with significantly higher prevalence of microcytic anaemia than their counterparts of other occupation. It is understandable that being jobless predisposes one to lower income and therefore inadequate financial resources to provide nutritious meals to meet the daily nutrient requirement of the household. However, children whose parents/guardians were fishermen and farmers were expected not to have microcytic anaemia because they have access to iron-rich food sources. Nevertheless, observations from this study, congruent to previous studies in this area [21, 34], show that many farmers do not consume the best of the foods they produce but rather sell them for money and consume the less presentable ones. Fish and vegetables are common sources of iron in the area which if consumed in the best state regularly alongside fruits will reduce the occurrence of anaemia. This reasserts reports from other studies [63, 64] that the low or nonconsumption of fruits, vegetables, and iron-rich animal sources increases risks for anaemia.

The overall low prevalence of malarial anaemia in this population (19.6%) reveals that malaria may not be a major contributor to the overall anaemia prevalence. This proportion is lower than the 27.7% previously observed in the same area [34]. Even though submicroscopic infection with *Plasmodium falciparum* infection has been associated with anaemia in other studies [65, 66] which was not investigated in the current study, the lack of association between malaria parasite density and anaemia likely highlights its limited contributions to the burden of anaemia in the study population. Of concern is the significant association of child's age, parent's age, education level, and occupation, with malarial anaemia in the regression analysis which may be directly linked to the influence of both malaria and anaemia. Febrility and malaria positivity influence on malarial anaemia prevalence cannot be overemphasized [21]. Nonetheless, fever, being a nonspecific symptom, may have also resulted from other infections which were not considered in this study.

While the findings of this study may be applicable in several areas in the region and elsewhere with similar environmental conditions and microclimates as well as cultural practices, there is a limitation in its applicability in areas nonendemic for malaria and having variable eating habits. However, the findings provide valuable information that could be used in the development of appropriate, context specific control measures against anaemia, microcytic anaemia, and malarial anaemia by public health authorities.

## 5. Conclusions

With anaemia prevalence still well above the cut-off value of 40%, it is important to reevaluate childhood determinants that foster its presence and also revisit the implementation strategies that have so far been put in place. An anaemia-monitoring system, especially those aimed at reducing nutritional anaemia, will effectively help in curbing anaemia. While microcytic anaemia is closely moving to the red zone as a public health problem in urban areas of Mount Cameroon, malarial anaemia is of mild public health concern. The high microcytic anaemia prevalence in children aged ≤5 years, those living at low altitude and within the community, shows that some insidious factors other than malaria are at work. While age, parent's/guardian's occupation and ethnicity, and moderate parasitaemia were risk factors for microcytic anaemia, malarial anaemia had as risk factors child's age, parent's age and occupation, and a ≤4 times weekly consumption of plantains. Therefore, when planning interventions to reduce anaemia prevalence in the community, strategies that will elevate the socioeconomic status of the parents should be integrated to aid better and healthy food choices to reduce anaemia due to nutritional deficiencies.

## Figures and Tables

**Figure 1:** Effect of age and parents' education level on dietary habits.

**Table 1:** Characteristics of the 566 participants enrolled in the study.

Parameter	Total
% (*n*)	100 (566)
*Gender*	
Female	52.8 (299)
Male	47.2 (267)
Age group in years	
1–5	51.4 (291)
6–10	24.9 (141)
11–15	23.7 (134)
Mean age (SD) in years	6.4 (4.5)
Mean height (SD) in cm	112.6 (28.4)
Mean weight (SD) in kg	23.7 (14.6)
Mean Hb conc. in g/dL	10.4 (2.0)
*Sociodemographic factors*	
Altitude of residence	
Lowland	61.5 (348)
Highland	38.5 (218)
Point of presentation	
Community	36.7(208)
Hospital	63.3 (358)
Health district	
Buea	37.5 (212)
Limbe	62.5 (354)
Age of household head (years)^a^	*N* = 407
≤25	3.9 (16)
26–35	28.5 (116)
36–50	44.2 (180)
>50	23.3 (95)
Education level of household head	
Primary	23.3 (132)
Secondary	40.6 (230)
Tertiary	31.6 (179)
No formal	4.4 (25)
Family size	
≤5	50.5 (286)
6–10	43.8 (248)
>10	5.7 (32)
*Clinical factors*	
Mean temperature (SD) in °C	37.1 (1.1)
Malaria parasite prevalence	27.7 (157)
Fever prevalence	27.7 (157)
Prevalence of inflammation	58.4 (211)
Anaemia prevalence	68.7 (389)
Microcytosis	48.9 (277)
Malnutrition	15.2 (86)

^a^Calculated for 407 participants.

**Table 2:** Prevalence of malaria parasite and malnutrition by sociodemographic factors.

Parameter	Category	*N*	Malaria parasite prevalence % (*n*)	*χ* ^2^,*P* value	Malnutrition prevalence	*χ* ^2^,*P* value
Gender	Male	267	28.5 (76)	0.133,	16.5 (44)	0.648,0.421
	Female	299	27.1 (81)	0.715	14.0 (42)	
Age	1–5	291	28.9 (84)	**11.855,0.003**	21.0 (61)	**17.110,<0.001**
	6–10	141	35.5 (50)		6.4 (9)	
	11–15	134	17.2 (23)		11.9 (16)	

Altitude	Lowland	348	32.8 (114)	**11.360,0.001**	18.1 (63)	**5.934**
	Highland	218	19.7 (43)		10.6 (23)	**0.015**

Point of presentation	Community	208	17.8 (37)	**16.243, <0.001**	17.8 (37)	1.717
	Hospital	358	33.5 (120)		13.7 (49)	0.190

Parents' age^c^	≤25	16	6.2 (1)	3.940,0.268	25.0 (4)	**5.076,0.166**
	26–35	116	22.4 (26)		17.2 (20)	
	36–50	180	20.6 (37)		13.9 (25)	
	>50	95	14.4 (14)		8.4 (8)	

Education	Primary	132	19.7 (26)	7.288,0.063	17.4 (23)	2.516,0.472
	Secondary	230	28.3 (65)		13.9 (32)	
	Tertiary	179	31.3 (56)		14.0 (25)	
	No formal	25	40.0 (10)		24.0 (6)	

Family size	1–5	286	32.5 (93)	**6.605,0.037**	13.6 (39)	2.629,0.269
	6–10	248	23.0 (57)		17.7 (44)	
	>10	32	21.9 (7)		9.4 (3)	

Occupation	Farming	123	29.3 (36)	11.239,0.081	10.6 (13)	**14.495,0.025**
	Civil servant	77	24.7 (19)		10.4 (8)	
	Petty trading	63	33.3 (21)		9.5 (6)	
	Private worker	92	20.7 (19)		16.3 (15)	
	Fishing	103	28.2 (29)		23.3 (24)	
	Jobless	69	39.1 (27)		23.2 (16)	
	Retired	39	15.4 (6)		10.3 (4)	

Ethnicity	Coastal	212	19.3 (41)	**2.861,0.581**	10.8 (23)	**10.816, 0.029**
	Grassland	112	17.0 (19)		12.5 (14)	
	Forest	5	20.0 (1)		20.0 (1)	
	Sahel	7	0.0 (0)		14.3 (1)	
	Other ethnic groups	68	23.5 (16)		26.5 (18)	

^c^Calculated for 407 participants. *P* values in bold are statistically significant.

**Table 3:** Prevalence of anaemia, microcytic anaemia, and malarial anaemia with respect to sociodemographic and clinical factors.

Parameter	Category	*N*		Prevalence [% (*n*)] of					
				Anaemia	*P* value	Microcytic anaemia	*P* value	Malarial anaemia	*P* value
*Sociodemographic factors*									
Gender	Male	267		70.0 (187)		39.7 (106)	0.196	20.6 (55)	
	Female	299		67.6 (202)	0.525	34.4 (103)		18.7 (56)	0.57.6
Age	1–5	291		69.1 (201)		43.3 (126)	**<0.001**	21.6 (63)	
	6–10	141		70.2 (99)	0.781	38.3 (54)		25.5(35)	
	11–15	134		66.4 (89)		21.6 (29)		9.0 (12)	**0.001**
Altitude	Lowland	348		77.3 (269)		49.1 (179)		24.4 (85)	
	Highland	218		55.0 (120)	**<0.001**	17.4 (38)	**<0.001**	11.9 (26)	**<0.001**
Point of presentation	Community	208		81.2 (169)		42.8 (89)		15.9 (33)	
	Hospital	358		61.5 (220)	**<0.001**	33.5 (120)	**0.028**	21.8 (78)	0.089
Parents' age^c^	≤25	16		68.8 (11)		12.5 (2)		6.2 (1)	
	26–35	116		80.2 (93)	**0.006**	39.7 (46)	**0.004**	21.6 (25)	**0.046**
	36–50	180		70.6 (127)		31.1 (56)		12.8 (23)	
	>50	95		57.9 (55)		18.9 (18)		9.5 (9)	
Family size	1–5	286		69.6 (199)		40.9 (117)		21.7 (62)	
	6–10	248		71.4 (177)	**0.002**	33.9 (84)	0.086	17.3 (43)	0.449
	>10	32		40.6 (13)		25.0 (8)		18.8 (6)	
Education	Primary	132		75.8 (100)		40.2 (53)		13.6 (18)	
	Secondary	230		73.5 (169)	**0.001**	39.1 (90)	0.306	20.9 (48)	0.057
	Tertiary	179		57.0 (102)		31.3 (56)		20.1 (36)	
	No formal	25		72.0 (18)		40.0 (10)		36.0 (9)	
Occupation	Farming	123		71.5 (88)		39.0 (48)		18.7 (23)	
	Civil servant	77		57.1 (44)		18.2 (14)		14.3 (11)	
	Petty trading	63		52.4 (33)		25.4 (16)		19.0 (12)	
	Private worker	92		76.1 (70)		35.9 (33)		16.3 (15)	
	Fishing	103		86.4 (89)	**<0.001**	56.3 (58)	**<0.001**	24.3 (25)	0.094
	Jobless	69		63.8 (44)		46.4 (32)		30.4 (21)	
	Retired	39		53.8 (21)		20.5 (8)		10.3 (4)	
Ethnicity	Coastal	212		68.9 (146)		27.8 (59)		12.7 (27)	
	Grassland	112		61.6 (69)		23.2 (26)		15.2 (17)	
	Forest	5		100.0 (5)	**0.002**	60.0 (3)	**0.002**	20.0 (1)	0.546
	Sahel	7		71.4 (5)		14.3 (1)		0.0 (0)	
	Other ethnic groups	68		88.2 (60)		48.5 (33)		19.1 (13)	

*Clinical factors*									
Fever	No		409	69.2 (283)		35.2 (144)		15.4 (63)	
	Yes		157	67.5 (106)	0.700	41.4 (65)	0.172	30.6 (48)	**<0.001**
Malaria parasite status	Positive		157	70.7 (111)		49.7 (78)		70.7 (111)	
	Negative		409	60.0 (278)	0.531	32.0 (131)	**<0.001**	0.0 (0)	**<0.001**
Parasite load	Low		92	70.7 (65)		50.0 (46)		70.7 (65)	
	Moderate		43	74.4 (32)	0.665	62.8 (27)	**0.009**	74.4 (32)	0.665
	High		22	63.6 (14)		22.7 (5)		63.3 (14)	
Malnutrition	No		480	11.3 (20)	0.082	14.6 (52)	0.586	14.7 (67)	0.529
	Yes		86	17.0 (66)		16.3 (34)		17.1 (19)	
Inflammation	No		150	67.3 (101)	**0.011**	44.7 (67)	0.436	22.7 (34)	0.902
	Yes		211	79.1 (167)		48.8 (103)		23.2 (49)	

^c^Calculated for 407 participants: *P* value obtained by *χ*^2^, *P* values in bold are statistically significant.

**Table 4:** Prevalence of anaemia, microcytic anaemia, and malarial anaemia with respect to nutritional status and dietary habits.

Parameter	Status	*N*	Prevalence [% (*n*)] of					
			Anaemia	*P* value	Microcytic anaemia	*P* value	Malarial anaemia	*P* value
Stunting	No	494	66.6 (329)		35.0 (173)		18.8 (93)	
	Yes	59	83.1 (49)	**0.010**	47.5 (28)	0.060	23.7 (14)	0.368
Underweight	No	405	67.9(275)		40.7 (165)		22.7 (92)	
	Yes	19	89.5 (17)	**0.047**	47.4 (9)	0.566	21.1 (4)	0.866
Wasting	No	249	67.5(168)		43.7 (107)		21.7 (54)	
	Yes	23	60.9 (14)	0.520	21.7 (5)	**0.048**	13.0 (3)	0.330
Hand washing before meal	Yes	352	68.8 (242)		28.4 (100)		13.6(48)	
	No/seldom	55	80.0 (44)	0.090	40.0 (22)	0.081	18.2 (10)	0.370
Daily meal	1	41	80.5 (33)		39.0 (16)		19.5 (8)	
	2	146	70.5 (103)		30.8 (45)		13.7 (20)	
	3	220	68.2 (150)	0.285	27.7 (61)	0.336	13.6 (30)	0.597
Weekly fruits consumption	1-2	173	74.6 (129)		28.9 (50)		15.6 (27)	
	3-4	57	57.9 (33)		31.6 (18)		14.0 (8)	
	>4	177	70.1 (124)	0.058	30.5 (54)	0.910	13.0 (23)	0.782
Weekly meat consumption	1-2	178	69.7 (124)		29.2 (52)		15.2 (27)	
	3-4	59	83.1 (49)		37.3 (22)		20.3 (12)	
	>4	170	66.5 (113)	0.054	28.2 (48)	0.407	11.2 (19)	0.199
Weekly plantain consumption	1-2	210	65.7 (138)		28.6 (60)		16.2 (34)	
	3-4	68	85.3 (58)		25.0 (17)		20.6 (14)	
	>4	129	69.8 (90)	**0.009**	34.9 (45)	0.289	7.8 (10)	**0.025**

*P* values in bold are statistically significant.

**Table 5:** Multinomial regression analysis examining sociodemographic, clinical, hygiene, and dietary factors associated with anaemia, microcytic anaemia, and malarial anaemia.

Parameter	Category	Anaemia		Microcytic anaemia		Malarial anaemia	
		AOR (95% CI)	*P* value	AOR (95% CI)	*P* value	AOR (95% CI)	*P* value
*Sociodemographic factors*							
Gender	Male	1.0 (0.6-1.6)	0.904	1.2 (0.7–2.0)	0.417	0.7 (0.4–1.4)	0.355
	Female	Reference		Reference		Reference	
Age	1–5	0.9(0.5–1.6)	0.685	2.4 (1.3–4.6)	**0.007**	1.9 (0.8–4.5	0.163
	6–10	1.1 (0.5–2.1)	0.852	2.0 (1.0–3.9)	0.060	3.3 (1.4–8.1)	**0.008**
	11–15	Reference		Reference		Ref	
Altitude	Lowland	4.0 (1.3–12.4)	**0.017**	1.7 (0.5–6.1)	0.401	3.3 (0.8–13.6)	0.096
	Highland	Reference		Reference	—	Reference	—
Presentation	Hospital	1.5 (0.5–4.4)	0.515	0.4 (0.1–1.4)	0.133	2.8 (0.7–11.5)	0.147
	Community	Reference	—	Reference	—	Reference	—
Family size	>10	0.2 (0.1–0.7)	**0.017**	1.2 (0.4–4.7)	0.748	1.0 (0.3–4.1)	0.979
	6–10	1.1 (0.6–1.8)	0.828	1.1(0.6–1.8)	0.833	0.8 (0.4–1.5)	0.446
	1–5	Reference		Reference	—	Reference	—
Parents' age	≤25	1.0 (0.3–3.7)	0.991	0.5 (0.1–2.4)	0.349	0.8 (0.1–7.1)	0.826
	26–35	1.8 (0.9–4.0)	0.117	1.7 (0.8–3.7)	0.163	2.6 (1.0–6.6)	**0.049**
	36–50	1.2 (0.6–2.2)	0.645	1.8 (0.9–3.8)	0.105	1.4 (0.6–3.4)	0.481
	>50	Reference	—	Reference	—	Reference	—
Education level	No formal	1.9 (0.6–5.7)	0.261	0.6 (0.2–1.8)	0.388	0.2 (0.1–0.6)	**0.005**
	Primary	1.5 (0.5–4.4)	0.506	0.5 (0.2–1.5)	0.215	0.2 (0.1–0.6)	**0.003**
	Secondary	1.1 (0.3–3.4)	0.902	0.5 (0.2–1.8)	0.303	0.3 (0.1–0.9)	**0.030**
	Tertiary	Reference	—	Reference	—	Reference	—
Ethnicity	Coastal	1.4 (0.4–5.5)	0.645	1.4 (0.4–4.3)	0.599	0.6 (0.3–1.3)	0.194
	Grassland	2.2 (0.6–8.5)	0.265	0.8 (0.3–2.5)	0.701	0.8 (0.3–1.7)	0.493
	Forest	—	—	15.7 (1.6–155.4)	**0.019**	1.1 (0.1–10.3)	0.961
	Sahel	4.3 (0.4–41.7)	0.210	0.1 (0.0–1.5)	0.098		—
	Others	Reference	—	Reference		Reference	—
Occupation	Farming	2.2 (1.0–4.5)	**0.042**	2.5 (1.1–5.9)	**0.038**	2.0 (0.7—6.2)	0.225
	Civil servant	1.1 (0.5–2.5)	0.735	0.9 (0.3–2.3)	0.762	1.5 (0.4–4.9)	0.543
	Petty trading	0.9 (0.4–2.1)	0.885	1.3 (0.5–3.5)	0.573	2.1 (0.6–56.9)	0.242
	Private worker	2.7 (1.2–6.0)	**0.013**	2.2 (0.9–5.3)	0.087	1.7 (0.5–5.5)	0.373
	Fishing	5.5 (2.3–12.7)	**<0.001**	0.3 (0.0–1.5)	**<0.001**	2.8 (0.9—8.7)	0.073
	Jobless	1.5 (0.7–3.4)	0.313	3.4 (1.4–8.3)	**0.009**	3.8 (1.2–12.1)	**0.023**
	Retired	Reference	—	Reference		Reference	—

*Clinical factors*							
Malnutrition	Yes	1.2 (0.1–31.4)	0.903	0.2 (0.0–2.3)	0.196	1.2 (0.0–31.4)	0.903
	No	Reference		Reference		Reference	
Stunting	Yes	0.4 (0.0–12.5)	0.621	7.9 (0.7–84.2)	0.088	0.4 (0.0–12.5)	0.621
	No	Reference		Reference		Reference	—
Underweight	Yes	0.7 (0.0–12.2)	0.831	2.3(0.6–9.5)	0.245	0.7 (0.0–12.2)	0.831
	No	Reference		Reference	—	Reference	—
Wasting	Yes	—	—	1.4 (0.1–12.2)	0.912	—	—
	No	Reference		Reference	—	Reference	—
Parasitaemia	High	0.3 (0.1–1.8)	0.183	0.1 (0.0–1.2)	0.071	0.1 (0.0–1.9)	0.129
	Moderate	0.2 (0.0–1.3)	0.086	2.6 (1.0–6.6)	**0.048**	0.9 (0.2–3.9)	0.932
	Low	Ref		Reference		Ref	
Inflammation	Yes	1.1 (0.3–4.3)	0.937	2.0(0.9–4.4)	0.084	1.1 (0.3–4.3)	0.937
	No	Ref		Ref		Ref	

*Dietary factors*							
Weekly fruit consumption	1-2	1.4 (0.8–2.4)	0.240	1.0 (0.6–1.7)	0.995	0.9 (0.5–1.9)	0.861
	3-4	0.4 (0.2–0.8)	**0.015**	1.1 (0.6–2.2)	0.783	0.7 (0.3–1.8)	0.471
	>4	Reference		Reference	—	Reference	—
Weakly meat consumption	1-2	1.2 (0.7–2.1)	0.430	1.1 (0.7–1.9)	0.661	1.3 (0.7–2.6)	0.436
	3-4	2.5 (1.1–5.6)	**0.026**	1.8 (0.9–3.6)	0.077	1.6 (0.7–3.8)	0.346
	>4	Reference		Reference	—	Reference	—
Weekly Plantain consumption	1-2	0.7 (0.4–1.2)	0.174	0.7 (0.2–1.2)	0.158	2.2 (1.0–4.8)	0.052
	3-4	2.5 (1.1–5.6)	**0.034**	0.5 (0.2–1.0)	0.057	2.9 (1.2–7.3)	**0.024**
	>4	Reference	—	Reference	—	Reference	

*P* values in bold are statistically significant.

## Data Availability

All the datasets generated and analysed during the current study are presented in the paper.
